# Cross-Cultural Adaptation and Reliability of the Home Falls and Accidents Screening Tool (HOME FAST) in Assessing Fall-Risk Home Hazards for Stroke Using Technologies over a Conventional Home Visit

**DOI:** 10.1155/2022/6044182

**Published:** 2022-03-16

**Authors:** Husna Ahmad Ainuddin, Muhammad Hibatullah Romli, Tengku Aizan Hamid, Mazatulfazura S. F. Salim, Hazwan Mat Din, Lynette Mackenzie

**Affiliations:** ^1^Department of Rehabilitation Medicine, Faculty of Medicine and Health Sciences, Universiti Putra Malaysia, 43400 Serdang, Selangor, Malaysia; ^2^Centre of Occupational Therapy Studies, Faculty of Health Sciences, Universiti Teknologi MARA, 42300 Puncak Alam Selangor, Malaysia; ^3^Department of Rehabilitation Medicine, Universiti Putra Malaysia Teaching Hospital, Universiti Putra Malaysia, 43400 Serdang, Selangor, Malaysia; ^4^Malaysian Research Institute on Ageing (MyAgeing), Universiti Putra Malaysia, 43400 Serdang, Selangor, Malaysia; ^5^Discipline of Occupational Therapy, School of Heath Sciences, Faculty of Medicine and Health, University of Sydney, Camperdown, NSW 2050, Australia

## Abstract

**Objective:**

This study is aimed at translating the Home Falls and Accidents Screening Tool (HOME FAST) into the three main languages spoken in Malaysia and investigating its reliability through an alternative technology-based evaluation.

**Methods:**

Translation into three languages and cross-cultural adaptation of the HOME FAST was conducted via the five steps adopted from the Mapi Institute. For interrater reliability, occupational therapists who attended a face-to-face home hazard workshop were recruited. Each therapist rated the HOME FAST by using the provided combination of videos and photographs of stroke survivors manoeuvring in their home. For test-retest reliability, the same occupational therapists were invited to rate the same combination of photographs and videos again. Reliability was analysed using Gwet's AC_1_ and Bland and Altman's plot to describe agreement.

**Results:**

The translation challenges were minimal and rectifiable. A Bahasa Melayu, Mandarin, and Tamil versions of the HOME FAST were developed. Overall interrater reliability for both video (AC_1_ = 0.91) and photograph (AC_1_ = 0.91) were good. The test-retest reliability yielded similar outcome (video: overall AC_1_ = 0.92 and photograph: overall AC_1_ = 0.93).

**Conclusion:**

Using alternative technology (video and photograph) to do a home hazard assessment was feasible. However, the asynchronous nature of these methods has limitations in clarifying certain aspects in the home. Moving forward, potential investigation on other technologies such as telehealth for synchronous and real-time interaction is warranted.

## 1. Introduction

Falls are a long-term complication after a stroke [1]. Chronic illnesses in aging populations may lead to a state of vulnerability and frailty [2], thus contributing to falls [3, 4]. Impairments in physical, cognitive, and psychological aspects due to stroke can increase the risk of falls [5]. A fall after a stroke could result in injuries, increase fear of falling, increase costs of care [6], and affect daily activities and independence as well as community participation [7], either during the acute [8] or chronic phases of a stroke [9]. Hence, poststroke falls are of great concern to both the individual and community at large [10].

Established risk factors for falls after stroke include poor functioning of activities of daily living (ADL), disease-related mental health factors, physical and sensory deficits, fear of falling, and having a history of falls [11–13]. When compared with studies of older people and falls, one neglected crucial risk factor of falls is environmental factors [14]. Home hazards in and around the house are recognized as one of the contributing factors to the risk of falls [15–17]. The use of instruments to identify home hazards has been well documented in the literature [18]. These instruments are used as part of fall prevention initiatives or to identify necessary modifications with the goal of encouraging the participation of older people in the community. However, many nonstandardised instruments are adopted to assess the home environment [19], and little evidence has been produced demonstrating the reliability of many standardised instruments [20] especially within stroke population.

An ideal screening practice involves a safe, practical, and cost-effective approach that is both valid and reliable [21] and encourages effort for early detection to determine the need for a more comprehensive intervention. The Home Falls and Accidents Screening Tool (HOME FAST) is a suitable instrument for the task as it has extensive evidence of validity and reliability [18]. The HOME FAST was created in Australia and has been used in fall prevention services, and it is aimed at identifying older persons living at home who have a risk of falling due to environmental conditions in and around their home [22]. The HOME FAST has been validated among the older population in several countries and has fair to excellent interrater and test-retest reliability [20, 23, 24]. The administration of the HOME FAST involves an on-site observation method conducted either by clinicians or by clients. The clinical utility of the HOME FAST, which requires self-training, is relatively generic, quick to administer, and makes it favourable to use in practice.

The challenge of doing a home hazard assessment is conducting the home visit. Factors such as clinical responsibilities, the time required for travel, lack of knowledge among practitioners, the client's lack of awareness about the purpose of a home visit and gaining permission, and the client's availability to observe the homes of clients hinder the practice of conducting a home visit [24, 25]. The issue is more significant for the stroke population, as prevention of falls is usually considered secondary to interventions for physical impairments [26]. There is also a misperception that physical improvement alone can progressively prevent falls [27]. Thus, home visit practices have been abandoned.

An alternative method is required to substitute a missing home visit assessment. Assessing home hazards via digital photographs and videos is a cost-effective technique [18]. Although there is limited research which demonstrates the use of digital photography to identify home hazards, it does provide an alternative to remotely examine the environment for fall-risk hazards [28–30]. Furthermore, video cameras are familiar to the majority of people and do not require substantial training, and some are designed for persons with limited technical skills [31]. To improve the use of standardised instruments in practice, it is recommended that the feasibility of using digital photographs [18, 32] or a video is determined to complement a home hazard assessment.

Standardised instruments to assess the risk of falls in Malaysian stroke survivors' homes are lacking [33], thus could lead to fall prevention programs being implemented based on inaccurate data. Many of the stroke population are older people, and Malaysia consists of three major ethnicities of Malay, Chinese, and Indian. Most older people in each ethnic group comprehend their own native language better [34], thus the need for cultural adaptation of the instruments. This study is aimed at translating the HOME FAST into Bahasa Melayu, Mandarin, and Tamil and establishing the reliability of the HOME FAST for stroke using technologies over a conventional face-to-face home visit.

## 2. Methods

### 2.1. Overview of Method

Translation of the HOME FAST into three languages and interrater reliability and test-retest reliability were examined. Procedures and results are described under each type of psychometric test. Approval was obtained from the Ethics Committee for Research Involving Human Subjects, Universiti Putra Malaysia (JKEUPM-2019-320), the National Stroke Association Malaysia, and the online Malaysian Stroke Survivors Support Group. Informed consent was obtained from the stroke participants and healthcare practitioners who agreed to participate in the study. All participants volunteered to participate and had the right to withdraw at any time during the study. A flowchart of the study is illustrated in Figure 1.

### 2.2. Instrument

The HOME FAST is a screening instrument that examines home hazards through the interaction of individuals and their home environment when performing activities that could put them at risk of falls [22]. The HOME FAST assesses hazards via 25 items on seven domains consisting of flooring, furniture, lighting, bathroom, storage, stairways/steps, and mobility. Each item in the HOME FAST is rated either “yes” (no hazards), “no” (hazardous), or “NA” (not applicable). The score is calculated by counting and totalling the “no” response, in which each response contributed 1 mark. The range of the score is from 0 to 25, and higher scores indicate more hazards at home, therefore a higher risk of falls [22]. The HOME FAST is administered via observation and interview of how the individual functions within their home environment [24]. It was designed in Australia but had been internationally adopted [24]. The HOME FAST has been validated among the older population in the community [20, 23] and can be self-administered by older people, multidisciplinary healthcare practitioners, and the public [24, 35].

### 2.3. Translation and Cross-cultural Adaptation

The Mapi Research Trust's five-stage recommendation which consists of translation, synthesis, back translation, clinical review, and cognitive debriefing was used as a guideline and to validate the cross-cultural adaptations of the instrument [36].

#### 2.3.1. Forward Translation and Synthesis

The purpose of the translation process was to produce a version of the HOME FAST in Bahasa Melayu, Mandarin, and Tamil with “conceptual, semantic, and operational equivalence” to the original Australian English version. The selection of the targeted language was due to the major ethnic composition of Malaysia, which is Malay, Chinese, and Indian [34]. A total of six translators (two bilingual translators for each language) who were native speakers of the respective languages and fluent in English translated the instrument. For every language version, one translator had a background in health and the other was a professional translator with a nonhealth background. The two translators worked independently without influencing each other's translation. The two drafts were then reconciled, and the researchers decided on which translation was more equivalent to the original meaning and appropriate for the language speakers. Single reconciled Bahasa Melayu, Mandarin, and Tamil versions were then finalised.

#### 2.3.2. Backward Translation

A backward translation of the finalised forward translations was obtained in the source language (Australian English) by a professional translator who was a native speaker of the respective language, fluent in English, and had no prior knowledge of the instrument. The backward translated version was compared with the original HOME FAST by a multidisciplinary team leading to the production of the second reconciled version in Bahasa Melayu, Mandarin, and Tamil. Similarly, translation inconsistencies and language concerns that developed during this procedure were rectified.

#### 2.3.3. Clinical Review and Cognitive Debriefing

A discussion was held with four physiotherapists, a speech therapist, and one occupational therapist to obtain feedback to be incorporated into the third reconciled version of HOME FAST. There are representative on each ethnicity in the discussion group. The Bahasa Melayu version was used as a reference as every Malaysian, regardless of ethnicity, understands Bahasa Melayu. Therefore, any discrepancy between Mandarin and Tamil was discussed and harmonized synchronously with the Bahasa Melayu version. Cognitive debriefing for the Bahasa Melayu version of the HOME FAST was conducted with three cognitively intact stroke survivors and three caregivers who took an average of about 20 minutes to complete the assessment. This was to ensure that the final versions of the questionnaire were comprehensible and acceptable, and that the language used was simple and suitable for the intended future users of the assessment. Face-to-face interviews were used for this preliminary test to obtain comments and suggestions on the scale from interviewees. The final reconciled Bahasa Melayu, Mandarin, and Tamil versions were produced based on the consultation from the clinicians and participants.

### 2.4. Interrater and Test-Retest Reliability

#### 2.4.1. Study Design and Participants

A cross-sectional study design was implemented, and two populations were recruited for the study: (i) stroke survivors having a home hazard evaluation via a face-to-face home visit and (ii) occupational therapists as the comparison raters. For a fair quality reliability analysis, a sample size of 30-50 paired home ratings was considered [39].

#### 2.4.2. Stroke Participants

Stroke participants were recruited from an online stroke survivors' support group and from two community-based stroke rehabilitation centres in the Klang Valley area. The inclusion criteria were as follows: (1) ≥21 years old, (2) diagnosis of unilateral hemispheric stroke according to the definition of the American Heart Association [37], (3) at any phases of the stroke, and (4) able to follow simple two-step instructions. Patients with unstable medical conditions, diagnosed with severe cognitive impairments, or aphasic (based on medical records) were excluded. Informed consent was obtained for all participants before conducting the home assessments. Convenience sampling was conducted to recruit participants. Stroke survivors were recruited at the selected National Stroke Association of Malaysia (NASAM) centres in Selangor and Kuala Lumpur. The screening was conducted using the Modified Rankin Scale (from no symptoms to moderately severe disability) via a face-to-face interview at the centre, and participants that fulfilled the inclusion criteria were invited to participate in the study. Written consent forms were documented before the participation of the participants. Only consenting stroke survivors were recruited for the study. Appointments for a home visit and assessment were set up by the researcher but the date and time were determined by the participants. The study was also advertised in the Malaysian Stroke Survivors Support Group with an invitation to participate in this study, and any group member who was interested was given instructions to contact the researchers. Once a group member had contacted the researcher, the researcher explained the study, asked for personal information, and established the functional status according to the Modified Rankin Scale via call, text, or WhatsApp. Once the participant fulfilled all the inclusion criteria, the information sheet and consent form together were given to the participant to sign. The researcher then made an appointment to conduct a home visit according to the date and time given by the participant.

#### 2.4.3. Comparison Raters

Occupational therapists were recruited as comparison raters. All raters were trained to administer and score the HOME FAST through a workshop, which comprised lectures and demonstrations, immediately before the reliability study. Administration and scoring procedures of the HOME FAST use the method described by Mackenzie et al. [22, 38] to ensure standardisation of data collection. Home hazard ratings from comparison raters were compared with a primary rater for interrater reliability.

#### 2.4.4. Procedures

The procedure for the reliability studies included the following:

*(1) Home Visit and Home Hazard Assessment*. The first author was also the primary rater for this study. On the day of the appointment for a home visit, the primary rater with a research assistant travelled to the participant's home. The primary rater explained the study to the stroke participant and conducted a manual on-site home hazard assessment. Following this, the research assistant recorded a video and captured a picture of key angles of the patient's home using a standard smartphone camera. At this point, the research assistant was not trained in the use of the HOME FAST and was simply capturing images of the home rather than the use of the home hazard assessment. The duration of this home visit was 1 hour for each home. The intention of not training the research assistant is to mimic lay people conducting the recording activity. All home visits were rated by the primary rater. In total, 18 homes were visited and evaluated. The data from the primary rater later became the baseline data for the comparison rater in the interrater reliability analysis.

*(2) Interrater Reliability*. A home hazard assessment workshop for the comparison raters was conducted at the researcher's university. Although all the comparison raters knew about the HOME FAST assessment, they did not have formal training prior to the workshop. A two and a half hours, face-to-face education and training workshop on the HOME FAST were conducted by the first and second authors. The background of the HOME FAST with detailed descriptions and administration was discussed in a 60-minute lecture. A 60-minute practical session later followed in which participants were asked to score the HOME FAST on their observation of a video and photographs of a person carrying out functional activities in the home environment [24]. The trainers scored the HOME FAST before conducting the workshop, and the scores were blinded to the raters. After the raters had finished evaluating the HOME FAST, a 30-minute discussion session was held in which the raters' results were compared to the trainers. Any discrepancies in the HOME FAST findings were then examined, and any queries were answered during that time.

After the training, these comparison raters were each given a set of the photographs and videos taken by the research assistant. The pair of photographs and video was randomly allocated for the raters. Photographs and video were accessed, and HOME FAST ratings were recorded via Google Form, on a computer at the university. Thus, the video and photographs were not downloaded or kept by the comparison raters. The comparison raters were given one hour to assess both the photographs and videos using the HOME FAST instrument. After the assessment was completed, all pictures and videos and the assessment results were collected for analysis. Additional comments and feedback on assessing home hazards via video and photographs were also recorded via an open-ended question on the Google Form after the assessment was completed.

*(3) Test-Retest Reliability*. For test-retest reliability, the same photographs and videos were reassessed by the same comparison raters after 18-76 days from the initial assessment. The duration is acceptable as there is no maturity bias that may occur due to the use of the same video but is long enough to prevent recall bias. The comparison raters were given an email link of the videos and a photograph of the home visits to reassess. The photographs and video were only able to be accessed electronically but were not able to be downloaded and kept.

#### 2.4.5. Data Analysis

The data analysis for this paper was generated by IBM SPSS version 26 and the Real Statistics Resource Pack software (Release 7.2) (Copyright 2013-2020) [40]. Descriptive statistics were used to summarize rater and stroke survivor characteristics, range, and distribution of the scores on the outcome measure. For both interrater and test-retest reliability, Gwet's AC_1_ is the statistic of choice for the case of two raters [41] Gwet's agreement coefficient can be used in more contexts than Kappa or Pi because it does not depend upon the assumption of independence between raters. The agreement value classifications are poor (AC_1_ ≤ 0), slight (AC_1_ = 0.01–0.20), fair (AC_1_ = 0.21–0.40), moderate (AC_1_ = 0.41–0.60), substantial (AC_1_ = 0.61–0.80), and almost perfect (AC_1_ = 0.81–1.00), based on the suggestion of Landis and Koch [42]. The Pearson correlation was applied for measuring the association between the two variables and ranges from -1 and 1, with 1(-1) indicating perfect positive (negative) correlation and 0 indicating no association between the variables [43].

The Bland-Altman plot method was used to examine the agreement between two raters in scoring the hazards for two parallel measurements [44]. This was generated by calculating the difference score between the comparison rater's score (*a*) and primary rater's score (*b*); (*a* − *b*) and the mean scores between the two raters (*a* + *b*)/2 and then plotting them against each other. When 95% of the mean scores fell within the boundaries of agreement, it was considered as an acceptable agreement between the two raters. The limits of agreement were generated by calculating the maximum limit from the mean difference ([*xa* + *xb*]/*x* + 1.96SD) and the minimum limit from the mean difference ([*xa* + *xb*]/*x* − 1.96SD). A positive mean difference meant the comparison rater had identified more hazards than the primary rater, and a negative mean difference implied vice versa, while for test-retest reliability, a positive mean indicates high hazard identification during the first assessment [24]. In addition, standard error of mean (SEM) was also calculated in order to determine an estimate of variability of possible values of means of samples [45]. It is projected that there will be less variability in the values of sample mean than in the initial population [45]. While there is no standard guideline for interpreting the SEM, however, smaller SEM value indicates a better interpretation.

## 3. Results

### 3.1. Translation and Cross-cultural Adaptation of the HOME FAST into the Three Languages

The adaptation and reliability testing process has produced a Bahasa Melayu, Mandarin, and Tamil versions of the HOME FAST. Several terms were challenging to be translated into the Bahasa Melayu. This could be seen during the forward translation process. These challenges arose either because of a lack of familiarity with Bahasa Melayu words that are rarely used in ordinary communication, or there are no direct or multiple translations available. These terms include “cords,” “floor coverings,” “non-slip,” “two doorways,” and “edge.” Harmonization on the most suitable terms to be used was conducted to produce the final forward translation of the HOME FAST Bahasa Melayu version. The backward translation of the Bahasa Melayu HOME FAST was conducted with ease as the terms selected during harmonization were appropriate and reflect the original English version of the HOME FAST. For the Mandarin and Tamil versions, the two languages were harmonized by two native speakers, respectively, who were Malaysian by cross-referencing the translation with the Bahasa Melayu and English versions. During the item evaluation process, no item was excluded from the original HOME FAST as all the items were considered by the clinicians as appropriate and relevant to the home environment and function of stroke survivors living in Malaysia. Furthermore, stroke survivors and caregivers during the cognitive interviews reported that the instrument was straightforward and easy to comprehend and utilise.

### 3.2. Reliability

A total of 18 stroke survivors and 20 healthcare practitioners participated in the interrater study. The mean age of stroke participants in the study was 57.5 years (SD = 14.57). More than half of the participants were male, and 72.2% were Malays; 50% of stroke survivors were retired or had no income, and 83.3% were more than 24 months poststroke. In all, 72.2% of participants reported a fall after stroke, and 44.4% lived with others in an apartment (Table 1). The first three stroke participants' videos taken had substantial missing components and could not be analysed while five videos were used for training purposes. In total, only 10 pairs of videos and photographs were rated by the comparison raters.

Twenty occupational therapists participated as a comparison rater and rated a total of 41 videos and photographs in the interrater study (Table 2). The mean age for interraters was 32.25 (±6.09). The same group of stroke participants was involved in the test-retest study; however, only 18 comparison raters (age mean: 31.22 ± 4.87) rated 37 pairs of videos and photographs of the HOME FAST in the test-retest study (Table 2). The set number of videos and photographs assessed by the comparison raters ranged from one to five with a median of two sets. When using digital photographs for assessment, a few therapists reported that the photographs did not capture the overall home hazards such as slippery floors and lighting at night.

#### 3.2.1. Interrater Reliability

*(1) Video*. The overall AC_1_ value for the video interrater reliability of the HOME FAST was 0.91 indicating good interrater reliability (95% CI: 0.74-0.98) (Table 3). The correlation between the primary rater and comparison raters was moderate (*r* = 0.48, *p* = 0.001). The mean of the HOME FAST score among comparison raters was 9.39 (95% CI, SD = 2.83, SEM = 0.44), and the mean for the HOME FAST score of the primary rater was 9.73 (95% CI, SD = 2.46, SEM = 0.38). The mean difference of 0.34 in the Bland and Altman graph plot in Figure 2 indicated that the primary rater identified more hazards compared to the comparison rater, and 95.1% of the difference score fell within the limits of agreement (95% CI, −4.98 to 5.66) which indicated consistency of the scoring.

*(2) Digital Photograph*. Meanwhile, the overall AC_1_ value for the interrater reliability of the HOME FAST of photographs was 0.91 indicating good interrater reliability (95% CI: 0.65-0.99) (Table 3). The correlation between the primary rater and comparison raters was *r* = 0.34, *p* = 0.03. The mean of the HOME FAST score among comparison raters was 9.83 (95% CI, SD = 3.15, SEM = 0.49), and the mean for the HOME FAST score of the primary-rater was 10.51 (95% CI, SD = 2.94, SEM = 0.46). The mean difference of 0.68 for the Bland and Altman in Figure 3 indicated that the primary rater identified more hazards compared to the comparison raters, and 95.1% of the difference score fell within the limits of agreement (95% CI, −6.18 to 7.54) indicating consistency of the scoring.

#### 3.2.2. Test-Retest Reliability

*(1) Video*. The mean interval time between the first and second assessments for the test-retest reliability study was 40.35 days. The overall AC_1_ value for the video test-retest reliability was 0.92 indicating satisfactory test-retest reliability (95% CI: 0.81-0.99) (Table 4). The correlation between the first and second assessments was *r* = 0.67, *p* < 0.001. The mean HOME FAST score for the first assessment was 9.62 (95% CI, SD = 2.78, SEM = 0.46), and for the second assessment was 8.54 (95% CI, SD = 2.73, SEM = 0.45). A positive mean difference was detected (*M* = 1.08) indicating raters identified more hazards on repeated than initial evaluations. However, 94.5% of the difference score fell between the limits of agreement (95% CI, −3.33 to 5.49), which is acceptable to be considered in which the comparison raters consistently scored the hazards over time as shown in Figure 4.

*(2) Digital Photograph*. The overall AC_1_ value for the photographs' test-retest reliability was 0.93 indicating satisfactory test-retest reliability (95% CI: 0.75-0.99) (Table 4). The mean HOME FAST score for photographs for the first assessment was 9.67 (95% CI, SD = 3.19, SEM = 0.53), and for the second assessment, it was 9.21 (95% CI, SD = 2.61, SEM = 0.43). The correlation between the first and second assessments was *r* = 0.49, *p* = 0.002. A slight positive mean difference (*M* = 0.46) indicated a minimal difference in hazard identification between the initial and repeated evaluations, and 100% of the difference score fell between the limits of agreement (95% CI, −5.37 to 6.29), which indicates the consistency of the comparison raters in scoring the hazards over time as shown in Figure 5.

## 4. Discussion

In this study, the translations were established while interrater and test-retest reliability of the HOME FAST in assessing fall-risk home hazards for stroke by using technologies over home visits via occupational therapists were evaluated. This prospective study revealed several promising findings.

### 4.1. Translation and Cross-cultural Adaptation of the HOME FAST

This is the first use of simultaneous multiple translation conducted in the cross-cultural validity of a home hazard assessment. This approach was found beneficial, effective in addition to time, and cost-saving. The initial translation was revised with the input of an expert panel to make it easier to read and comprehend, as well as to ensure language and cultural applicability in the Malaysian context [46]. The challenge in translation is evident for occupational therapy-use assessments but can be rectified similar with other studies in Malaysian context [47–49].

### 4.2. Reliability of the HOME FAST

The use of digital photography and video captured most of the environmental and functional elements identified by the HOME FAST. Its high acceptability and satisfactory ratings by occupational therapists make using technology to assess home hazards a feasible option.

The interrater reliability for using both a video and a set of photographs to evaluate home hazards via the HOME FAST among occupational therapists in this present study was satisfactory. The results are consistent with other studies that have reported similar trends of interrater reliability of home hazard assessments among occupational therapists [38, 50], performed consistently or better when compared with other screening tools that adopted technology [28–30] and among patients with dementia [51].

Most of the comparison raters identified a lower number of hazards compared with the primary rater, which is also supported by previous studies [20, 24]. This may be due to the primary rater having more experience in scoring criteria and interpretation of the HOME FAST items [24]. Furthermore, the primary rater scored the HOME FAST via an on-site home visit and thus may have a better representation of the hazards available. The results of the video and photograph test-retest reliability of the HOME FAST were also interpreted as satisfactory and were consistent with previous findings [24, 38, 50]. The test-retest reliability produced better results as the comparison raters had gained experience in scoring the HOME FAST during the interrater stage [24].

### 4.3. Evaluation of the HOME FAST via Technology

Recent studies have established the use of digital photographs and video as a means for home hazard assessment [28, 29, 31]. Occupational therapists administered the HOME FAST via assessing the videos and digital photographs provided. Thus, the overall assessment was based on judgment and clinical reasoning of the videos and photographs. Some therapists mention that a few of the digital photographs did not capture crucial angles that could provide them with specific information to assist in evaluating the home hazards. As the HOME FAST is a checklist for screening, the videos and photographs were taken with consideration of the research assistant and her understanding of the important aspects of the home that needs to be captured. This may have led to therapists not being able to assess beyond the images and could lead to assumptions when assessing. Providing the guideline early (for example, only the questions of the HOME FAST) to the client or responsible person to capture the photographs or video may be helpful to give some idea on what to expect [29]. Furthermore, using cameras with wide-angle lenses is helpful to improve the detection rate and validity [29].

The low score in interrater reliability of “outdoor paths” and “outdoor lighting” for the HOME FAST could be due to video and photograph-taking in broad daylight with the lights on. This is due to the therapist's difficulty in interpreting the situation at night, which necessitates the evaluations be made based on the lighting during daytime. For a more comprehensive assessment, a follow-up video or photograph would be required to be taken during the night as it would illustrate a better picture of the home environment. In contrast, a study by Daniel et al. [29] reported low agreement on pathways and slippery surfaces as it was difficult to identify slippery surfaces by photographing them. Furthermore, photographs did not always capture the whole room and thus obstructed pathways were often missed in the evaluation [29]. The supplementing via additional photographs for each section of the home is recommended as it could also provide more information for assessment [28]. The use of telehealth could also be suggested as it delivers a real-time, synchronous home safety evaluation and provides direct opportunity for clarification by the assessor to ask question to the client [52].

Given that this study was conducted in Malaysia, differences in culture and the terms of the hazards may also impede the agreement among comparison raters on the HOME FAST items [24]. For example, most homes do not have a bathtub, and this could give the understanding that it could be substituted with a shower/bathing area instead. Besides evaluating the physical environment and a person's physical function, attention to footwear (textured insoles, footwear modifications, and habitual footwear) is also important as it is a modifiable risk factor in falls prevention [53]. Nonetheless, the HOME FAST has demonstrated satisfactory interrater reliability in this study.

### 4.4. Limitation

The study indeed has some limitations. First, cognitive interviews were not carried out comprehensively for the Mandarin and Tamil languages. However, feedback received from the Bahasa Melayu version was incorporated for the other two languages in the final versions. Second, the generalisability of the study findings is limited, given the sample size of the study and the study being conducted in an urban area only. However, this study did demonstrate proof of principle, suggesting that using technology to assess HOME FAST should be further validated in different settings which could include both clinical and community settings with larger sample sizes. Finally, the comparison raters were exclusively occupational therapists, which has limited the generalisability of findings to other health professional groups. Future studies should investigate the use of technology in assessing HOME FAST with different client populations.

## 5. Conclusion

Using alternative methods to do a home hazard assessment is demonstrably feasible. However, some limitations are pertinent whereby technology is unable to capture overall home situations. A brief protocol should be developed to enhance the implementation of using the video and photographs in assessing home hazards. Future studies should investigate synchronous and real-time technology such as telehealth.

## Figures and Tables

**Figure 1:** Flowchart of study.

**Figure 2:** Bland-Altman plot for interrater reliability (video).

**Figure 3:** Bland-Altman lot for interrater reliability (photograph).

**Figure 4:** Bland-Altman plot for test-retest reliability (video).

**Figure 5:** Bland-Altman plot for test-retest reliability (photograph).

**Table 1:** Demographics of stroke participants (*N* = 18).

Characteristic		Mean (±SD)	*N* (%)
Age		57.67 (±14.57)	

Gender	Male		11 (61.1)
	Female		7 (38.9)

Race	Malay		14 (77.8)
	Chinese		4 (22.2)
	Indian		0 (0)

Marital status	Married		15 (83.3)
	Widower/divorced		3 (16.7)

Monthly household income	B40 (<RM6180)		9 (50.0)
	M40 (RM6180–RM12470)		8 (44.4)
	T20 (>RM12470)		1 (5.6)

Type of house	Apartment/condominium		8 (44.4)
	One-storey landed		3 (16.7)
	Double/multistorey landed		7 (38.9)

Home modification^∗^	Yes		7 (38.9)
	No		11 (61.1)

Months poststroke	<24 months		3 (16.7)
	≥24 months		15 (83.3)

Affect body side	Right		11 (61.1)
	Left		7 (38.9)

Walking aid use	Yes		10 (55.6)
	No		8 (44.4)

Falls after stroke	Yes		13 (72.2)
	No		5 (27.8)

Location of falls	Indoor		7 (53.8)
	Outdoor		5 (38.5)
	Both		1 (7.7)

Activity when falling	Walking		6 (46.2)
	Transfer		1 (7.7)
	Toileting/showering		1 (7.7)
	Standing		5 (38.4)

^∗^Includes installation of grab bar, the use of a shower seat, tape for carpet, antislip tape for stairs, antislip mat in bathrooms, and the use of assistive devices.

**Table 2:** Demographics of comparison raters for interrater and test-retest reliability.

Characteristic		Interrater (*N* = 20)	Test-retest (*N* = 18)
		*n* (%)	*n* (%)
Gender	Male	6 (30.0)	4 (22.2)
	Female	14 (70.0)	14 (77.8)

Race	Malay	18 (90.0)	17 (94.4)
	Others	2 (20.0)	1 (5.6)

Highest education level	Diploma	7 (35.0)	6 (33.3)
	Bachelor	4 (20.0)	4 (22.2)
	Master	7 (35.0)	6 (33.3)
	Doctorate	2 (10.0)	2 (11.1)

Type of work	Public	17 (85.0)	16 (88.9)
	Private	3 (15.0)	2 (11.1)

Work setting	Clinical	13 (65.0)	11 (61.1)
	Community	2 (10.0)	2 (11.1)
	Education	5 (25.5)	5 (27.8)

Work experience	<1 year	1 (5.0)	1 (5.6)
	1-5 years	7 (35.0)	7 (38.9)
	6-10 years	5 (25.0)	4 (22.2)
	>10 years	7 (35)	6 (33.3)

Experience conducting home assessment	<1 year	6 (30.0)	6 (33.3)
	1-5 years	8 (40.0)	7 (38.9)
	6-10 years	5 (25.0)	5 (27.8)
	>10 years	1 (5.0)	0 (0)

**Table 3:** Interrater agreement of HOME FAST on video and photographs evaluation.

HOMEFAST item	Video			Photograph		
	AC_1_	Quality	%	AC_1_	Quality	%
Walkway cluttered	0.96	Almost perfect	78.0	0.90	Almost perfect	58.5
Poor condition of floor coverings	0.93	Almost perfect	65.9	0.93	Almost perfect	68.3
Slippery floor surfaces	0.92	Almost perfect	58.5	0.90	Almost perfect	53.7
Loose mats	0.93	Almost perfect	68.3	0.91	Almost perfect	61.0
Difficulty with bed transfers	0.95	Almost perfect	85.4	0.93	Almost perfect	73.2
Difficulty with lounge transfers	0.92	Almost perfect	73.2	0.85	Almost perfect	53.7
Poor lighting	0.94	Almost perfect	65.9	0.97	Almost perfect	87.5
No access to bedside light	0.98	Almost perfect	90.2	0.98	Almost perfect	92.3
Poor lighting on outdoor paths	0.77	Substantial	64.1	0.78	Substantial	57.5
Difficulty with toilet transfers	0.89	Almost perfect	63.4	0.90	Almost perfect	65.9
Difficulty with bath transfers	0.90	Almost perfect	82.9	0.94	Almost perfect	85.4
Difficulty with shower transfers	0.89	Almost perfect	78.0	0.91	Almost perfect	63.4
No access to grab rails in bath	0.98	Almost perfect	92.7	0.99	Almost perfect	90.2
No slip-resistant mats in bathroom	0.96	Almost perfect	80.5	0.97	Almost perfect	87.8
Toilet not near to bedroom	0.96	Almost perfect	87.8	0.91	Almost perfect	58.5
Difficulty reaching items in kitchen	0.93	Almost perfect	65.9	0.92	Almost perfect	63.4
Difficulty carrying meals	0.95	Almost perfect	68.3	0.95	Almost perfect	75.6
Inadequate/absent steps/stair rails indoor	0.87	Almost perfect	80.5	0.95	Almost perfect	95.1
Inadequate/absent steps/stair rails outdoor	0.85	Almost perfect	53.7	0.86	Almost perfect	73.2
Using stairs	0.84	Almost perfect	75.6	0.96	Almost perfect	87.8
Undefined stair edges	0.91	Almost perfect	82.5	0.96	Almost perfect	92.7
Entrance doors	0.97	Almost perfect	72.5	0.95	Almost perfect	65.0
Outdoor paths	0.74	Substantial	61.0	0.65	Moderate	46.3
Improper footwear	0.97	Almost perfect	85.4	0.96	Almost perfect	82.9
Hazardous pets	0.93	Almost perfect	87.8	0.96	Almost perfect	87.8

Note. AC_1_: Gwet's AC_1_ analysis; %: agreement percentage.

**Table 4:** Findings on the test-retest reliability of HOME FAST video and photographs.

HOMEFAST item	Video			Photograph		
	AC_1_	Quality	%	AC_1_	Quality	%
Walkway cluttered	0.94	Almost perfect	75.7	0.90	Almost perfect	56.8
Poor condition of floor coverings	0.90	Almost perfect	56.8	0.96	Almost perfect	81.1
Slippery floor surfaces	0.90	Almost perfect	56.8	0.94	Almost perfect	73.0
Loose mats	0.95	Almost perfect	75.7	0.89	Almost perfect	78.4
Difficulty with bed transfers	0.95	Almost perfect	75.7	0.96	Almost perfect	83.8
Difficulty with lounge transfers	0.91	Almost perfect	75.7	0.94	Almost perfect	81.1
Poor lighting	0.96	Almost perfect	78.4	0.97	Almost perfect	80.6
No access to bedside light	0.98	Almost perfect	89.2	0.97	Almost perfect	85.7
Poor lighting on outdoor paths	0.81	Substantial	68.6	0.84	Almost perfect	69.4
Difficulty with toilet transfers	0.85	Almost perfect	70.3	0.93	Almost perfect	67.6
Difficulty with bath transfers	0.94	Almost perfect	81.1	0.90	Almost perfect	78.4
Difficulty with shower transfers	0.95	Almost perfect	78.4	0.86	Almost perfect	59.5
No access to grab rails in bath	0.99	Almost perfect	94.6	0.99	Almost perfect	97.3
No slip-resistant mats in bathroom	0.97	Almost perfect	81.1	0.98	Almost perfect	91.9
Toilet not near to bedroom	0.97	Almost perfect	86.5	0.98	Almost perfect	83.8
Difficulty reaching items in kitchen	0.95	Almost perfect	75.7	0.94	Almost perfect	73.0
Difficulty carrying meals	0.96	Almost perfect	83.8	0.96	Almost perfect	83.8
Inadequate/absent steps/stair rails indoor	0.88	Almost perfect	83.8	0.95	Almost perfect	91.9
Inadequate/absent steps/stair rails outdoor	0.98	Almost perfect	91.9	0.92	Almost perfect	89.2
Using stairs	0.82	Almost perfect	73.0	0.94	Almost perfect	81.1
Undefined stair edges	0.90	Almost perfect	77.8	0.95	Almost perfect	89.2
Entrance doors	0.98	Almost perfect	91.7	0.98	Almost perfect	86.1
Outdoor paths	0.82	Almost perfect	70.3	0.75	Substantial	64.9
Improper footwear	0.96	Almost perfect	78.4	0.98	Almost perfect	86.5
Hazardous pets	0.98	Almost perfect	94.6	0.97	Almost perfect	89.2

Note. AC_1_: Gwet's AC_1_ analysis; %: agreement percentage.

## Data Availability

The data used to support the findings of this study are available from the corresponding author upon request.
